RETRACTED

# Thoracoscopic Lobectomy versus Segmentectomy in the Treatment of Patients with Early-Stage Lung Cancer

**DOI:** 10.1155/2022/4376968

**Published:** 2022-05-06

**Authors:** Chuankui Li, Xiaoxiao Ma, Yifan Yang, Qicai Li, Haiwei Sang, Guowen Wang, Tao Tao, Zuyi Wang

**Affiliations:** Department of Thoracic Surgery, The First Affiliated Hospital of Bengbu Medical College, Bengbu, Anhui 233000, China

## Abstract

**Objective:**

To assess the clinical efficacy of thoracoscopic lobectomy and segmentectomy in the treatment of patients with early-stage lung cancer.

**Methods:**

A total of 70 patients with early-stage non-small cell lung cancer who were treated in our hospital from April 2018 to May 2020 were recruited and assigned at a ratio of 1 : 1 to receive either segmentectomy (observation group) or lobectomy (control group). Outcome measures included clinical efficacy, surgery-related indicators, pulmonary function indicators (forced vital capacity (FVC) and forced expiratory volume in one second (FEV1)), postoperative complications, and recurrence and metastasis.

**Results:**

There was no significant difference in the clinical efficacy between the two groups (*P* > 0.05). Segmentectomy was associated with a longer operation time and shorter hospital stay compared to lobectomy (*P* < 0.05). There was no statistical significance in the amount of intraoperative blood loss and the number of lymph nodes dissected (*P* > 0.05). Segmentectomy resulted in significantly higher FVC and FEV1 levels in patients compared to lobectomy (*P* < 0.05). There was no significant difference in the incidence of postoperative complications between the two groups (*P* > 0.05). The two groups of patients were followed up for 12 months after the operation, and there was no recurrence or metastasis in either group.

**Conclusion:**

The two surgical methods have similar efficacy and safety profiles, but for the treatment of patients with early-stage lung cancer, thoracoscopic segmentectomy is associated with a shorter hospital stay and better protection of the lung function of patients compared to lobectomy.

## 1. Introduction

Lung cancer is currently the malignant tumor with highest morbidity and mortality worldwide. In recent years, the incidence of lung cancer and its related deaths in China has been increasing year by year [1]. Non-small cell lung cancer accounts for about 78% of all lung cancer cases and is characterized by slow spread and low sensitivity to radiotherapy and chemotherapy, resulting in poor clinical efficacy of radiotherapy and chemotherapy in patients with non-small cell lung cancer [2]. Clinically, surgery is the mainstay of treatment for non-small cell lung cancer. Surgery can effectively relieve clinical symptoms, reduce body pain, and improve the prognosis of patients [3]. Lobectomy combined with mediastinal lymph node dissection is the standard surgical procedure for the clinical treatment of early-stage non-small cell lung cancer. It can completely remove the tumor and achieve a promising clinical curative effect [4]. However, with the promotion of clinical minimally invasive surgery, the operation of early-stage non-small cell lung cancer requires the preservation of the normal lung tissue to a maximum extent, to better preserve the lung function and enhance the postoperative quality of life of patients [5]. Wang et al. [6] have shown that thoracoscopic segmentectomy for patients with early-stage non-small cell lung cancer can preserve the healthy lung tissue to a greater extent than thoracoscopic lobectomy. In the present study, 70 patients with early-stage non-small cell lung cancer who were treated in our hospital from April 2018 to May 2020 were recruited to analyze and compare the clinical efficacy of thoracoscopic lobectomy versus segmentectomy in the treatment of patients with early-stage lung cancer.

RETRACTED

## 2. Materials and Methods

### 2.1. Baseline Data

A total of 70 patients with early stage nonsmall cell lung cancer who were treated in our hospital from April 2018 to May 2020 were recruited and assigned at a ratio of 1 : 1 to receive either segmentectomy (observation group) or lobectomy (control group). There were 19 males and 16 females in the observation group, aged 23–78 years, with an average age of (50.34 ± 7.27) years; 15 cases of left lung tumors and 20 cases of right lung tumors; tumor size of (≤30) mm; 21 cases of carcinoma in situ, 13 cases of adenocarcinoma, 1 case of squamous carcinoma; 6 cases of left upper lung apicoposterior segment, 5 cases of left lower lung dorsal segment, 4 cases of left upper lobe lingual segment, 3 cases of right upper lung anterior segment, 4 cases of right lower lung dorsal segment, 5 cases of right upper lung tip segment, and 4 cases of posterior segment of the right upper lung. In the control group, there were 18 males and 17 females; aged 23–71 years, with an average age of (50.18 ± 7.09) years; 17 cases of left lung tumor and 18 cases of a right lung tumor; tumor size of (≤30) mm; 19 cases of adenocarcinoma in situ, 12 cases of adenocarcinoma, and 4 cases of squamous cell carcinoma; 10 cases of left upper lobe lobectomy, 7 cases of left lower lobe lobectomy, 12 cases of right upper lobe lobectomy and 6 cases of right lower lobe lobectomy. The research was approved by the Ethics Committee of the First Affiliated Hospital of Bengbu Medical College, no. B2U991.

RETRACTED

### 2.2. Inclusion and Exclusion Criteria

Inclusion criteria are as follows: (1) the preoperative imaging diagnosis was T1N0M0, and the tumor diameter was within 3 cm; (2) aged 20–80 years old; (3) diagnosis conforming to the diagnostic criteria of nonsmall cell lung cancer in nonsmall cell lung cancer; (4) no radio therapy and chemotherapy before surgery; (5) all patients were diagnosed by X-ray, CT, MRI, and pathological biopsy; (6) lesions <5 cm and no distant metastases on imaging; and (7) lesions extending to ≥1 adjacent lung segment and complete resection achieved by anatomical lung segment. Exclusion criteria are as follows: (1) pregnant or lactating women; (2) other lung diseases; (3) other systemic tumor diseases; and (4) incomplete clinical data.

### 2.3. Methods

The patients in the observation group received thoracoscopic segmentectomy. With the patient in the decubitus position, after general anesthesia, the one-port or two-port method was adopted. A thoracoscope was placed through the main port, and a wedge-shaped lung resection was performed under the thoracoscope. The resected tissue samples were sent for rapid cryopathological examination during the operation. The dissection started at the root of the lung segment and deepened in the same direction, gradually exposing the superficial segmental blood vessels and segmental bronchi in the surgical field, and the connection between the lung segments was dissected. Prior to clipping the segmental bronchus, the anesthesiologist assisted in the expansion of the lung to confirm that the clipped bronchus is the target bronchus. The intersegmental fissure was excised using a thoracoscopic incision stapler. During the operation, lymph node sampling was performed at the same time and sent for rapid cryopathological examination. If the pathological results indicated the presence of lymph node metastasis, lobectomy was performed.

The patients in the control group received thoracoscopic lobectomy. The operation position, anesthesia method, and operation ports were the same as those in the observation group. Before the operation, the chemical glue was injected next to the tumor under the guidance of CT to locate the tumor. The resected nodules were sent for rapid cryopathological examination during the operation. The bronchus, pulmonary vein, pulmonary artery, and dysplastic interlobar fissure were severed using a linear cutting and stapler, and the lobe where the lesion was located was resected. Routine systematic dissection of hilar and mediastinal lymph nodes was performed.

### 2.4. Outcome Measures

(1) Efficacy criteria: at the 4th week after treatment, short-term efficacy was evaluated with reference to the efficacy evaluation criteria for solid tumors: complete remission (CR)—the lesions disappeared and lasted for at least 4 weeks; partial remission (PR)—the tumor in patients was reduced by >50%, which lasted for at least 4 weeks; stable disease (SD)—the tumor increased by less than 25% or reduced by <50%; progressive disease (PD)—the tumor increased by >25%. Treatment response rate (RR) = CR rate + PR rate; disease control rate (DCR) = CR rate + PR rate + SD rate. (2) Operation-related indicators: operation time, intraoperative blood loss, hospital stay, and the number of lymph node dissections were recorded. (3) Pulmonary function indicators: the two groups of patients were tested for routine pulmonary function using a pulmonary function tester before and 3 months after surgery. The pulmonary functions included forced vital capacity (FVC) and forced expiratory volume in one second (FEV1). (4) The medical staff in our hospital recorded the postoperative complications of the two groups of patients. The postoperative complications included pulmonary infection, atelectasis, air leakage, and arrhythmia. (5) The patients were followed up for 12 months to record the recurrence and metastasis.

RETRACTED

### 2.5. Statistical Analysis

All data analyses were performed with SPSS 21.0 software. The measurement data were expressed as (*x* ± *s*) and analyzed using the independent samples *t*-test. Count data were expressed as the number of cases (rate) and examined by the *X*^2^ test. Differences were considered statistically significant at *P* < 0.05.

## 3. Results

### 3.1. Baseline Data

There was no significant difference in general data such as gender, age, lesion location, and tumor size between the two groups, as shown in Table 1.

### 3.2. Clinical Efficacy

There was no significant difference in clinical efficacy between the two groups (*P* > 0.05, Table 2).

### 3.3. Surgery-Related Indicators

Segmentectomy was associated with a longer operation time and shorter hospital stay compared to lobectomy (*P* < 0.05). There was no statistical significance in the amount of surgical blood loss and the number of lymph nodes dissected (*P* > 0.05) (Table 3).

### 3.4. Pulmonary Function Indicators

Segmentectomy resulted in significantly higher FVC and FEV1 levels in patients compared to lobectomy (*P* < 0.05) as shown in Table 4.

### 3.5. Postoperative Complications

There was no significant difference in the incidence of postoperative complications between the two groups (*P* > 0.05), as shown in Table 5.

### 3.6. Postoperative Follow-Up

The two groups of patients were followed up for 12 months after the operation, and there was no recurrence or metastasis in either group.

RETRACTED

## 4. Discussion

Lobectomy is considered the standard surgical treatment for early-stage non-small cell lung cancer [7]. However, in recent years, the academic research community has put forward different views on the treatment of early-stage non-small cell lung cancer, as early-stage non-small cell lung cancer is associated with different degrees of functional decline in the patient's body, and the underlying diseases of the patient may complicate the treatment [8]. In recent years, a growing body of evidence has shown that there is no significant difference in the long-term efficacy between segmentectomy and lobectomy in the treatment of patients with early-stage non-small cell lung cancer. Seguin-Givelet et al. [9] studied 247 patients with early-stage non-small cell lung cancer who underwent thoracoscopic segmentectomy or lobectomy and found that patients who received either treatment of the two surgical methods had a 10-year disease-free survival, and there was no significant difference in duration and overall survival [10]. The non-small cell lung cancer guidelines also encourage hospitals that meet their conditions to selectively perform segmentectomy for patients with early-stage non-small cell lung cancer [11].

Pulmonary segmentectomy has been rapidly developed in recent years. The strict clinical indications for surgery and the strict requirements for operator proficiency and overall cooperation of the anesthesia team have hindered the clinical application of segmentectomy. There have been controversies about the effectiveness of segmentectomy in the treatment efficacy and the preservation of lung function; however, segmentectomy is mainly indicated for lung cancer patients with poor cardiopulmonary function that is not suitable for lobectomy, poor physical condition, or previous lobectomy. Overseas clinical research has shown that there is no significant difference in clinical outcomes between lobectomy and segmentectomy in a retrospective cohort study of patients with clinical stage I non-small cell lung cancer, and similar results have been obtained in other similar studies [12]. The results showed that there was no significant difference in the treatment efficacy between the two groups of patients. There was no significant difference in the short-term efficacy of segmentectomy in patients with early-stage non-small cell lung cancer. Moreover, segmentectomy was associated with a longer operation time and shorter hospital stay compared to lobectomy; there was no statistical significance in the comparison of the amount of surgical blood loss and the number of lymph nodes dissected between the two groups of patients. The results of surgery-related indexes were similar to those reported in previous studies. The reason may be that, in the early stage of non-small cells, segmentectomy causes less trauma to the patient [12]. The operation time of segmentectomy is relatively longer, which is attributed to the deep location of segmental bronchi and blood vessels and the difficulty of their exposure for resection [13]. Segmentectomy contributes more to the preservation of the lung tissue of the patient compared to lobectomy, thereby promoting the postoperative recovery of the patient and shortening the length of hospital stay [14].

RETRACTED

Here, there was no significant difference in the number of lymph nodes dissected between the two surgical methods, and there has been no clinical consensus on whether intersegmental lymph node dissection should be performed after segmentectomy. The cryopathological results of intraoperative sampling of hilar or mediastinal lymph nodes were negative, and the probability of intersegmental lymph node metastasis was only 0.5%, suggesting that intersegmental lymph node dissection is not clinically necessary. In the present study, specific dissection of intersegmental lymph nodes was skipped. Lobectomy was adopted only in the case of positive cryopathological results. Zhang et al. [15] found that segmentectomy can better preserve the lung function of patients with early-stage non-small cell lung cancer. Furthermore, segmentectomy herein resulted in significantly higher FVC and FEV1 levels of patients compared to lobectomy (*P* < 0.05), suggesting a better outcome of segmentectomy in preserving the lung function of patients compared to lobectomy [16, 17].

Moreover, after lobectomy, the remaining lobe on the ipsilateral side will compensatively expand, shift, and compress the bronchi, which increases the risk of airway resistance and reduces pulmonary ventilation [18]. The results of the present study showed that there was no statistical significance in the incidence of postoperative complications between the two groups of patients. The safety of treatment in patients with early-stage non-small cell lung cancer is also reliable [19]. The results showed that there was no recurrence or metastasis in the two groups of patients during the 12-month follow-up [20].

Patients with lung cancer mostly have Qi and Yin deficiency, and the administration of prescriptions to benefit Qi and nourish Yin can regulate the internal environment of the body, improve the immunity of the body, and reduce the toxic reactions of chemotherapy and radiotherapy [6]. Chinese medicine applied in the treatment of lung cancer can be used as a complementary method to western medicine treatment and plays an important role in controlling lesions and improving symptoms for patients who are considered inoperable. However, there are still some problems and shortcomings in the treatment of bronchial lung cancer with TCM to be addressed, which require more in-depth research.

RETRACTED

## 5. Conclusion

Segmentectomy and lobectomy have similar efficacy and safety profiles, but for the treatment of patients with early-stage lung cancer, thoracoscopic segmentectomy is associated with a shorter hospital stay and better protection of the lung function of patients compared to thoracoscopic lobectomy.

## Figures and Tables

**Table 1:** Baseline data (*n* (%)).

	Observation group (*n* = 35)	Control group (*n* = 35)	*t*/*x*^2^	*P*
Gender			0.057	0.811
Male	19	18		
Female	16	17		
Pathological type				
Carcinoma in situ	21	19		
Adenocarcinoma	13	12		
Squamous carcinoma	1	4		
Mean age (year)	50.34 ± 7.27	50.18 ± 7.09	0.093	0.926
Lesion site			0.516	0.473
Left	15	17		
Right	20	18		
Size (mm)	13.76 ± 2.14	13.88 ± 2.26	−0.228	0.82

**Table 2:** Comparison of efficacy (*n* (%)).

	Observation group (*n* = 35)	Control group (*n* = 35)	*x* ^2^	*P*
CR	16	15		
PR	11	12		
SD	4	3		
PD	4	5		
RR	27 (77%)	27 (77%)	0.0	1.0
DCR	31 (89%)	30 (86%)	0.128	0.721

**Table 3:** Comparison of surgery-related indicators (*x* ± *s*).

Groups	*n*	Operation time (min)	Intraoperative blood loss (mL)	Postoperative hospital stay (d)	Number of lymph nodes dissected (*n*)
Observation group	35	138.53 ± 33.49	95.16 ± 15.32	5.83 ± 1.15	12.27 ± 2.38
Control group	35	112.61 ± 28.56	100.47 ± 17.58	6.89 ± 1.41	12.19 ± 2.23
*t*	—	3.484	−1.347	−3.447	0.145
*P*	—	0.001	0.182	0.001	0.885

**Table 4:** Comparison of pulmonary function indexes (*x* ± *s*).

Groups	*n*	FVC (%)		FEV1 (%)	
		Before	After	Before	After
Observation group	35	2.87 ± 0.45	1.96 ± 0.37	2.12 ± 0.44	1.69 ± 0.38
Control group	35	2.91 ± 0.50	1.53 ± 0.31	2.15 ± 0.48	1.29 ± 0.33
*t*	—	−0.352	5.27	−0.273	4.702
*P*	—	0.726	＜0.001	0.786	＜0.001

**Table 5:** Comparison of complications (*n* (%)).

	Observation group (*n* = 35)	Control group (*n* = 35)	*x* ^2^	*P*
Lung infection	2	1		
Atelectasis	1	0		
Air leak	1	1		
Arrhythmia	1	2		
Total (%)	5 (14%)	4 (11%)	0.128	0.721

## Data Availability

No data were used to support this study.
